RETRACTED

# A Novel Alkaloid from Marine-Derived Actinomycete *Streptomyces xinghaiensis* with Broad-Spectrum Antibacterial and Cytotoxic Activities

**DOI:** 10.1371/journal.pone.0075994

**Published:** 2013-10-01

**Authors:** Wence Jiao, Fenghua Zhang, Xinqing Zhao, Jiehan Hu, Joo-Won Suh

**Affiliations:** 1 School of Life Science and Biotechnology, Dalian University of Technology, Dalian, China; 2 First Affiliated Hospital of Dalian Medical University, Dalian, China; 3 Dalian Institute of Chemical Physics, Chinese Academy of Sciences, Dalian, China; 4 Division of Bioscience and Bioinformatics, Myongji University, Yongin, Korea; University Paris South, France

## Abstract

Due to the increasing emergence of drug-resistant bacteria and tumor cell lines, novel antibiotics with antibacterial and cytotoxic activities are urgently needed. Marine actinobacteria are rich sources of novel antibiotics, and here we report the discovery of a novel alkaloid, xinghaiamine A, from a marine-derived actinomycete *Streptomyces xinghaiensis* NRRL B24674^T^. Xinghaiamine A was purified from the fermentation broth, and its structure was elucidated based on extensive spectroscopic analysis, including 1D and 2D NMR spectrum as well as mass spectrometry. Xinghaiamine A was identified to be a novel alkaloid with highly symmetric structure on the basis of sulfoxide functional group, and sulfoxide containing compound has so far never been reported in microorganisms. Biological assays revealed that xinghaiamine A exhibited broad-spectrum antibacterial activities to both Gram-negative persistent hospital pathogens (e.g. *Acinetobacter baumannii*, *Pseudomonas aeruginosa* and *Escherichia coli*) and Gram-positive ones, which include *Staphylococcus aureus* and *Bacillus subtilis*. In addition, xinghaiamine A also exhibited potent cytotoxic activity to human cancer cell lines of MCF-7 and U-937 with the IC_50_ of 0.6 and 0.5 µM, respectively.

## Introduction

The increasing prevalence of infections caused by multi-drug-resistant (MDR) bacterial pathogens has aroused worldwide concern. In addition to methicillin-resistant *Staphylococcus aureus* (MRSA) and *Pseudomonas aeruginosa* strains which have caused serious healthcare-associated and community-onset infections [1], [2], *Acinetobacter baumannii* has received increasing attention recently as a persistent hospital pathogens due to the rapidly increasing number of infections among compromised and injured patients and the global spread of strains with resistance to multiple antibiotics [3], [4]. However, studies on novel antibiotics to treat drug resistant *A. baumannii* are still very limited [5]. Therefore, there is an urgent need to seek for new antibiotics for clinical infections caused by the MDR bacterial pathogens.

RETRACTED

Marine-derived actinomycetes are rich sources of novel secondary metabolites which harbour unique structures and have diverse biological activities such as antimicrobial, antitumor and immunosuppressive activities [6]–[8]. The obligate marine genera *Salinispora* and *Marinispora* have been characterized [9], [10], and structurally unique and biologically active secondary metabolites have been isolated, such as salinosporamide A with excellent cytotoxicity from *S. tropica* CNB-392 and marinomycins A with strong antimicrobial and cytotoxic activities from *Marinispora* sp. CNQ-140 [11]–[13]. Marine-derived streptomycetes are also widely studied as novel antibiotic producers, where interesting compounds with antibacterial activities and anticancer activities were reported to be isolated [14], [15].

In our previous studies, a marine-derived actinobacterium *Streptomyces xinghaiensis* was identified to be a new species, which was proved to exhibit broad-spectrum antibacterial activities [16]. Herein, we report the isolation, structure elucidation, and biological activities of a new compound with promising activities against various bacterial pathogens, including the two notorious opportunistic pathogens *A. baumannii* and *P. aeruginosa*. To our knowledge, the sulfoxide functional group-containing compound has so far never been observed in microorganisms.

## Materials and Methods

### Ethics statement

The clinical methicillin-resistant *S. aureus* (5301, 5438 and 5885) and *A. baumannii* used as test strains were isolated from the sputum samples of patients and provided by the First Affiliated Hospital of Dalian Medical University. The study and protocols using the bacterial strains from patients were approved by the Ethics Committee of First Affiliated Hospital of Dalian Medical University, China. The Ethics Committee of First Affiliated Hospital of Dalian Medical University waived the need for a written informed consent.

### Microbial strains and culture media

*S. xinghaiensis* was preserved in our lab as a glycerol stock at −80°C and also at China General Microbiological Culture Collection centre (CGMCC) with accession number of CGMCC 2251. *S. aureus* (CGMCC 1.89), *B. subtilis* (CGMCC 1.73), *E. coli* (CGMCC 1.797), *P. aeruginosa* (CGMCC 1.2031) and *C. albicans* (CGMCC 2.538) were used as test strains. The clinical isolates including strains *S. aureus* (5301, 5438 and 5885) and *A. baumannii* used as test strains were isolated from the sputum samples of patients, and the procedure used for strain isolation was approved by the Ethics Committee of the First Affiliated Hospital of Dalian Medical University. The Ethics Committee of First Affiliated Hospital of Dalian Medical University waived the need for a written informed consent. Bacteria and yeast strain were maintained on Luria Bertani (LB, tryptone 10 g/l, yeast extract 5 g/l, NaCl 10 g/l) and Yeast Extract Peptone Dextrose (YPD, yeast extract 5 g/l, peptone 10 g/l, glucose 20 g/l) slants at 4°C, respectively. The solid medium were prepared by adding 1.5% agar into the liquid media.

RETRACTED

*S. xinghaiensis* was activated in Tryptic Soytone Broth (TSB, BD Difco™) seed medium and the production medium was optimized based on the medium described by Wang et al [17], and was prepared as follows: soluble starch 20 g/l, soybean powder 25 g/l, (NH_4_)_2_SO_4_ 2 g/l, NaCl 2 g/l, K_2_HPO_4_ 0.5 g/l and CaCO_3_ 5 g/l. The medium was prepared with distilled water, and the pH was adjusted to 7.0 prior to sterilization.

### Cell lines

Four human cancer cell lines for cytotoxicity assays were purchased from the Committee of Type Culture Collection of the Chinese Academy of Sciences (CTCCCAS, Shanghai, China). The accession numbers of human breast cancer cells line MCF-7, human live cancer cell line SMMC-7721, human acute myelogenous leukemia cell line U-937 and human small cell lung cancer cell line NCI-H1688 are TCHu 74, TCHu 52, TCHu159 and TCHu154, respectively. All the cell lines were maitained in RPMI-1640 medium (Invitrogen) supplemented with 10% fetal bovine serum and cultured at 37°C in humidified air containing 5% CO_2_.

### Culture conditions of *S. xinghaiensis*

The fresh culture of *S. xinghaiensis* from the TSB agar plate was inoculated into 250 ml shaker flask with 50 ml TSB medium and cultivated at 30°C at 200 rpm for two days. The seed cultures were then inoculated into the production medium (200 ml medium in 500 ml shake flasks) with an inoculation rate of 10% and cultured at 30°C at 200 rpm for 9 days. Three percent resin HP-20 (w/v) was added into the production medium at the 3rd day after inoculation to improve the production of antibiotics.

### General experimental procedures

Optical rotations were determined with a JASCO P-1020 digital polarimeter. The ultraviolet (UV) data were obtained on a HP8453 spectrophotometer. Thermo Nicolet spectrometer was used for scanning IR spectroscopy. Electrospray ionization (ESI) spectra in both positive and negative ion modes were measured on a HP1100 LC-MS spectrometer. High-resolution-electrospray-ionization mass spectra (HR-ESIMS) were performed on a Q-TOF Micro Mass Spectrometer. ^1^H NMR, ^13^C NMR, DEPT135, HSQC and HMBC spectra were recorded on a Bruker Advance DPX400 spectrometer (400 and 100 MHz for ^1^H and ^13^C NMR, respectively) using tetramethylsilane (TMS) as an internal standard. Elemental analysis was performed on Vario EL ΙΙΙ (Elementar, Germany).

RETRACTED

### Extraction and isolation of antibacterial compounds

The fermentation broth (4 L) including both mycelia and resins was directly mixed with two volumes of methanol (MeOH) and was shaken at 150 rpm for 120 min to extract the bioactive compounds. Then the mixture was centrifuged at 5000 rpm for 10 min, after which the supernatant was concentrated under reduced pressure to obtainan aqueous solution. The aqueous solution was subsequently extracted three times with two volumes of ethyl acetate (EtOAC) and concentrated under reduced pressure to give a crude extract (10 g).

The crude extract was firstly analyzed using a HPLC system (Waters, USA) equipped with a Waters Symmetry C18 column (4.6 mm×250 mm, 5 µm). The mobile phase consisted of H_2_O/acetonitrile (ACN) with 0.1% TFA added to both solvents and a gradient elution step was applied as follows: 0–15 min, 5–100% ACN; 15–25 min, 100% ACN. The flow rate was 0.85 ml/min and the elution was monitored by the UV absorption at 254 nm.

The crude extract was then subjected to column chromatography (CC) over silica gel (300–400 mesh, Qingdao Marine Chemical Factory, Qingdao, China), and eluted with stepwise gradients of CH_2_Cl_2_, EtOAC and MeOH (100% CH_2_Cl_2_, CH_2_Cl_2_/EtOAc 2∶1, CH_2_Cl_2_/EtOAc 1∶1, CH_2_Cl_2_/EtOAc 1∶2, 100% EtOAc, EtOAc/MeOH 2∶1, EtOAc/MeOH 1∶1, EtOAc/MeOH 1∶2, and finally 100% MeOH, v/v), respectively, to obtain nine fractions (Fr.01-Fr.09). Bioassay-guided fractionation of the crude extract revealed that the antibacterial compounds against *S. aureus* existed in fractions Fr.04, Fr.06, Fr.07 and Fr.09 (174.3, 250.3, 186.5 and 145.7 mg, respectively), which were then fractionated by flash C18 column chromatography eluting with 30%, 60%, 80% and 100% MeOH/water mixtures to give several sub-fractions. The sub-fractions (Fr.04-2, Fr.06-3, Fr.07-2 and Fr.09-4) containing antibacterial compounds were then further purified by semi-preparative reversed-phase HPLC equipped with C18 column (Waters Symmetry Prep™ C18 7.8 mm×300 mm, 7 µm, 3 ml/min) to give compound E (named later as xinghaiamine A), D1, D2, D3, C1, C2, B1 and B2 (For detailed isolation procedure, see Fig. S1).

#### Xinghaiamine A

Brown, viscous oil; [α]_D_^20^+10.8° (c 0.245, MeOH); UV (MeOH) λmax (log ε) 232.5 (3.88), 295.3 (1.15), 320.6 (0.08) nm; IR (MeOH) λmax 2924, 2852, 1725, 1656, 1561, 1465, 1382, 1280, 1233, 1082 cm^−1^; ^1^H and ^13^C NMR, see Table 1; positive ESIMS showed a [M+Na]^+^ peak at m/z 747.5 and a [M-H]^+^ peak at *m/z* 723.2; HR-ESIMS m/z 747.3390 ([M+Na]^+^, calcd 747.3385 for C_50_H_48_N_2_OSNa).

RETRACTED

**Table 1:** NMR spectroscopic data (CD_3_OD) of xinghaiamine A^a^

Position	δ_C_, type	δ_H_ (*J* in Hz)	^1^H-^1^H cosy	HMBC
1	107.7 CH	6.46, s	3	3, 5, 9
2	143.2 C			
3	108.3 CH	6.76, m	1	1, 5, 11
4	138.3 C			
5	120.4 C			
6	134.5 C			
7	120.0 CH	8.17, m	9	5, 9, 12, 19
8	140.2 C			
9	116.1 CH	8.15, s	7	1, 5, 7, 19
10	122.2 C			
11	120.7 CH	7.28, m	12	3, 5, 6
12	125.8 CH	7.28, m	11	4, 5, 7
13	27.2 CH_2_	1.80, m	14	15, 21, 23, 24
14	27.5 CH_2_	1.92, m	13, 15	22, 23
15	53.4 CH	3.09, t (8)	14, 23	2, 13, 18, 22
16	51.8 CH_2_	2.85, t (8)	17	2, 18
17	22.3 CH_2_	1.49, m	16	19, 21, 23
18	37.1 C			
19	37.1 C			
20	28.8 CH_2_	1.29, s		8, 18, 22, 25
21	61.2 C			
22	34.3 C			
23	24.8 CH	2.12, d (12)	15	13, 14, 19, 21
24	20.9 CH_3_	1.33, s		13, 21, 23
25	17.3 CH_3_	1.23, s		8, 18, 20

a Data was recorded in CD_3_OD, 400 MHz for ^1^H-NMR and 100 MHz for ^13^C-NMR. The signals were assigned in combination with ^1^H-^1^H COSY, HSQC and HMBC.

### Biological activity assays

Antimicrobial activities of xinghaiamine A against *S. aureus* (CGMCC 1.89), *B. subtilis* (CGMCC 1.73), *E. coli* (CGMCC 1.797), *P. aeruginosa* (CGMCC 1.2031), *C. albicans* (CGMCC 2.538) and methicillin-resistant *S. aureus* (MRSA 5301, 5438 and 5885) as well as *A. baumannii* were investigated. Xinghaiamine A was dissolved in MeOH to test the MIC (minimal inhibitory concentration, defined as the lowest concentration of xinghaiamine A inhibiting visible growth of test strains) values, which were achieved using the method as described previously [18]. Tetracycline and vancomycin were employed as positive controls for the model strains and MRSA isolates respectively and MeOH was employed as the negative control.

The *in vitro* cytotoxic activities of xinghaiamine A against MCF-7, SMMC-7721, U-937 and NCI-H1688 were evaluated using the MTT (Methyl-Thiazol-Tetrozolium) method [19]. Briefly, 200 µL of cell suspension was inoculated to 96-well plates with a final concentration of 10^5^ cells/ml and cultured for 24 h. After that, 50 µl of xinghaiamine A dissolved in DMSO adjusted to various concentrations was added to each well. After the exposure to xinghaiamine A for 48 h, 20 µL of 5 mg/ml MTT solution was added to each well, and the plates were incubated for 4 h at 37°C. Then, 150 µl of DMSO was added in each well. The absorbance caused by formazan crystallization was recorded at 550 nm using scanning mutiwell spectrophotometer. The measurements were repeated for three times, and average value was obtained. The cell viability was calculated using the following formula: cell viability (%)  =  (OD_550 nm_ of the group treated with xinghaiamine A/OD_550 nm_ of the untreated group) ×100%. Cisplatin and DMSO were employed as positive and negative control, respectively.

RETRACTED

## Results

### Analysis of fermentation crude extract

The crude extract was analyzed by HPLC and it was found that compounds with retention time at 11.18, 11.32, 11.62, 12.16, 13.36, 13.62, 13.92 and 16.64 min may belong to the same family due to the similar UV absorption (Fig. 1), which we successively named B1, B2, C1, C2, D1, D2, D3 and E, temporarily. To evaluate the antibacterial activity of these compounds, a pre-bioassay was performed by collecting samples every minute and employing *S. aureus* as an indicator after about 20 mg crude extract was subjected to the analytical HPLC. The results indicated that the antibacterial activities of *S. xinghaiensis* were mainly due to this compound family, especially compound E, which we named xinghaiamine A and it exhibited antibacterial activity against *S. aureus* and was more easily purified. Thus we subsequently focused on this compound in the large scale isolation and purification.

**Figure 1:** Production of a family of compounds with unique UV spectra by *S. xinghaiensis*. 1a , HPLC profile of fermentation crude extract produced by *S. xinghaiensis*. The elution was monitored at 254 nm at a flow rate of 0.85 ml/min. **1b**, UV absorption of the compound family. Compound E was named as xinghaiamine A.

### Structural analysis of xinghaiamine A

Xinghaiamine A was isolated as brown viscous oil. The positive- and negative-ion mode ESIMS analysis of xinghaiamine A (*m/z* 747.5 [M+Na]^+^; *m/z* 723.2 [M-H]^+^) indicated a molecular weight of 724 Da (Fig. S2). The positive-ion mode HR-ESIMS data of xinghaiamine A exhibited a [M+Na]^+^ molecular ion peak at *m/z* 747.3390 (calculated 747.3385) consistent with the molecular formula of C_50_H_48_N_2_OS, requiring 27 degrees of unsaturation (Fig. S3). The characteristic absorption bands at 232, 295, and 320 nm of UV spectra demonstrated that a conjugated naphthalene ring chromophore (maxima at 218, 261, and 331 nm) was involved in xinghaiamine A. The IR absorption band at 1082 cm^−1^ suggested the presence of sulfoxide functional group (Fig. S4), which was also supported by a sulfur content of 4.3% in the elemental analysis result (Fig. S10). The ^13^C NMR spectrum (Table 1) in combination with the DEPT135 experiments and 2D NMR spectra possessed 25 carbon signals, including two methyls, five methylenes, eight methines, and ten quaternary carbons, which revealed a highly symmetric molecular structure of xinghaiamine A on the basis of sulfoxide moiety.

All of the protons were assigned to carbons by HSQC experiments. For each part, an interpretation of ^13^C NMR and DEPT spectrum data showed the aromatic part has twelve carbons, including six methines and six quaternary carbons, accounting for ten out of fourteen degrees of unsaturation. Further interpretation of ^1^H NMR spectrum of xinghaiamine A accounts for six aromatic protons at δ6.46 (s), 6.76 (m), 7.29 (m), 7.27 (m), 8.15 (s), and 8.17 (m). Analysis of NMR with both COSY (H1/H3, H7/H9, H11/H12) and HMBC spectrum (H1 to C3, H1 to C5, H1 to C9, H3 to C1, H3 to C5, H3 to C11, H7 to C5, H7 to C9, H7 to C12, H7 to C19, H9 to C1, H9 to C5, H9 to C7, H9 to C19, H11 to C3, H11 to C5, H11 to C6, H12 to C4, H11 to C5, H12 to C7) showed correlations which illustrated that these proton and carbon signals were components of a naphthalene ring substituted at the position of C-2, C-8 and C-4, C-6 (conjugate ring), respectively.

RETRACTED

The remaining aliphatic fragment requiring the other five sites of unsaturation was deduced to have five or four rings by sharing a ring with the aromatic portion. An interpretation of ^13^C NMR and DEPT spectroscopic data showed that the aliphatic part had thirteen carbons and eighteen protons, indicative of two methyls, five methylenes, two methines, and four quaternary carbons (Table 1). The δC 37.1 (C-19,-C) and δC 140.2 (C-8, -C) were established to be at the junction of the aromatic and aliphatic fragment by the HMBC correlations from H-20 to C-8, H-25 to C-8, H-7 to C-19 as well as H-9 to C-19. Also, the HMBC correlations from H-15 and H-16 to C-2 proved that C-2 was substituted with N. Obviously, the proton signals at δH 3.09 (C-15, -CH) and δH 2.85 (C-16, -CH_2_) were connected to N with a relative low magnetic field. The ^1^H-^1^H COSY cross peaks of H-13/H-14, H-14/H-15 and H-16/H-17 suggested that δH 1.80 (C-13, -CH_2_) and δH 3.09 (C-15, -CH) were linked to δH 1.92 (C-14, -CH_2_), δH 1.49 (C-17 -CH_2_) was linked to δ2.85 (C-16, -CH_2_), respectively. δC 61.2 (C-21,-C) was established to be linked with the sulfoxide moiety due to the unique lowest chemical shift in aliphatic fragment, which was also consistent with the characteristic of sulfoxide functional group. The structure of other aliphatic fragment was established on the basis of ^1^H-^1^H cosy (H15/H23) and HMBC correlations of (See Table 1, Fig. 2, 3 and Fig. S5, S6, S7, S8, S9).

**Figure 2:** Proposed chemical structure of xinghaiamine A.

**Figure 3:** Selected ^1^H-^1^H COSY (bold lines) and HMBC (red arrows) correlations of xinghaiamine A.

### Antimicrobial tests

Xinghaiamine A showed broad-spectrum antibacterial activities against several test strains. It exhibited superior antibacterial activity to *S. aureus*, *B. subtilis*, *E. coli*, and *A. baumanii* with the MIC values of 0.69, 0.35 0.17, 2.76 and 11.04 µM, respectively, which were much lower than those of tetracycline. However, the inhibition of xinghaiamine A to *P. aeruginosa* was not as good as that of tetracycline. Xinghaiamine A also showed considerable activities to the clinical MRSA isolates with MIC values of 2.76 and 5.52 µM, albeit not so good as the powerful antibiotic vancomycin. The inhibition to the pathogenic bacteria and clinical MRSA isolates of xinghaiamine A demonstrated that it has the potential to be an effective antibiotic to deal with the multi-drug resistant pathogens, especially *S. aureus* and *A. baumanii*. No obvious antifungal activity to *C. albicans* of xinghaiamine A was found when it was tested at concentrations up to 176.64 µM (Table 2).

RETRACTED

**Table 2:** Antimicrobial activities of xinghaiamine A (MIC, µM) against the test strains.

	MIC (µM)^a^		
	xinghaiamine A^b^	tetracycline^c^	vancomycin^c^
*S. aureus*	0.69	4.50	−^d^
*B. subtilis*	0.35	2.25	−
*E. coli*	0.17	1.13	−
*A. baumanii*	2.76	9.0	−
*P. aeruginosa*	11.04	4.50	−
*C. albicans*	>176.64	−	−
MRSA 5301	5.52	−	0.35
MRSA 5438	2.76	−	0.18
MRSA 5885	5.52	−	0.70

**a** MIC represented the lowest compound concentration apparently inhibiting microorganism growth. **b** Xinghaiamine A was dissolved in MeOH for MIC test and MeOH was used as the negative control. **c** Tetracycline and vancomycin were employed as positive controls for the pathogenic bacteria (*S. aureus*, *B. subtilis*, *E. coli*, *A. baumanii* and *P. aeruginosa*) and clinical MRSA isolates (5301, 5438 and 5885), respectively. d “−” indicated that the positive control was not measured for the test strains.

### *In vitro* cytotoxicity assays

*In vitro* cytotoxicity assays of xinghaiamine A against four human cancer cell lines revealed that xinghaiamine A exhibited considerable broad-spectrum anti-proliferative activities (Table 3). Of the four cell lines, superior activity of xinghaiamine A against U-937 was observed, with the minimum IC_50_ value of 0.5 µM. Good cytotoxic activities of xinghaiamine A were also observed agaist MCF-7 and NCI-H1688, with the IC_50_ values much lower than that of the control. In contrast, comparable activity against SMMC-7721 of xinghaiamina A and cisplatin was observed (Table 3).

**Table 3:** *In vitro* cytotoxicity of xinghaiamine A (IC_50_ µM) against four human cancer cell lines.

	Cytotoxicity (IC_50_,µM)			
	MCF-7	SMMC-7721	U-937	NCI-H1688
Xinghaiamine A^a^	0.6	6.3	0.5	2.2
Cisplatin^b^	4.2	8.5	13.5	14.6

**a** Xinghaiamine A was dissolved in DMSO for the IC_50_ test and DMSO was used as the negative control. **b** Cisplatin was employed as positive control for the human tumor cell lines.

RETRACTED

## Discussion

The sulfoxide containing natural products are very limited in nature, and the current naturally occurred sulfoxide compounds are commonly peptide derivatives from terrestrial plants including Brussels sprouts (*S*-methyl-cysteine sulfoxide) [20], and *Allium siculums* (*S*-alk(en)yl-L-cysteine sulfoxide, *S*-n-butyl-cysteine sulfoxide) [21]-[23], as well as rare marine secondary metabolites from marine invertebrates (marine sponge *Pseudoceratina purpurea*, ascidian *Polycitor* sp., etc.), which include psammaplin N, eudistomin K, lehualides J, varacins B and D, eudistomidin E and aplisulfamines [24]–[29]. However, so far no sulfoxide antibiotic has been reported to be produced by microorganisms. The sulfoxide moiety presented in xinghaiamine A is unprecedented in metabolites from marine actinomycete. Sulfoxide compounds have broad-spectrum of biological activities, including excellent antimicrobial, pesticidic and antitumor activities, and chemical synthesis of sulfoxide compounds also has aroused the interests of researchers [30]. The discovery of xinghaiamine A as the first sulfoxide compound from marine *Streptomyces* sp. also promotes the idea that the sulfoxide compounds from marine invertebrates may also have a microbial origin.

Xinghaiamine A exhibited broad-spectrum antibacterial activities against various tested strains, including *A. baumanii*, which remains one of the major multiply resistant bacterial pathogens for serious healthcare-associated and community-onset infections. The isolation of xinghaiamine A seems to provide powerful potential to combat the emergence of multi-drug-resistant microbial pathogens. In addition, compared with cisplatin, xinghaiamine A also displayed promising cytotoxic activities against a series of human cancer cell lines. Recently, the rapid development of resistance to multiple drugs in tumor chemotherapy has urged for the searching for novel drugs and the results above revealed that xinghaiamine A could be a potential clinically useful antitumor drug to combat with the increasing multi-drug resistant cancer cell lines, and the current study provided basis for further develop this novel compound for anticancer therapy.

## Supporting Information

Figure S1 **Flow chart of isolation and purification of antibacterial compounds from** ***S. xinghaiensis*** **.**
(TIF)

Figure S2 **ESI-MS spectrum of xinghaiamine A, (a) positive-ion mode (b) negative-ion mode.**
(TIF)

Figure S3 **Positive ion mode of HR-ESIMS spectrum of xinghaiamine A.**
(TIF)

Figure S4 **IR spectrum of xinghaiamine A.**
(TIF)

Figure S5 **^13^C NMR and DEPT135 spectrum of xinghaiamine A.** Compound was dissolved in CH_3_OD and data was recorded on a Bruker Advance DPX400 spectrometer of 400 MHz for ^13^C NMR using TMS as internal standard.
(TIF)

Figure S6 **^1^H NMR spectrum of xinghaiamine A.** Compound was dissolved in CH_3_OD and data was recorded on a Bruker Advance DPX400 spectrometer of 100 MHz for ^1^H NMR using TMS as internal standard.
(TIF)

Figure S7 **^1^H-^1^H COSY spectrum of xinghaiamine A.**
(TIF)

Figure S8 **HSQC spectrum of xinghaiamine A.**
(TIF)

Figure S9 **HMBC spectrum of xinghaiamine A.**
(TIF)

Figure S10 **Elementary analysis of xinghaiamine A.** The experiments were performed twice which were described as E1 and E2, respectively.
(TIF)
